The article "Medical Sports Data Privacy Protection Method Based on Legal Risk Control" was published in 2021. Journal: J Healthc Eng.

# Medical Sports Data Privacy Protection Method Based on Legal Risk Control

**DOI:** 10.1155/2021/6630429

**Published:** 2021-05-08

**Authors:** Liqiang Jia, Wei Fan

**Affiliations:** ^1^Department of Physical Education, East China University of Political Science and Law, Shanghai 201620, China; ^2^Department of Physical Education, Shanghai University of Political Science and Law, Shanghai 201701, China

## Abstract

With the continuous development of computer and network technology, the amount of information storage in medical information system is more and more large, which is prone to the problem of privacy information leakage, resulting in irreparable harm. In order to solve the problem of privacy leakage in the medical environment, a new privacy rating method is proposed according to the actual situation of the medical environment. The big data technology is used to effectively mine, analyze, integrate, and reuse medical data, and a new improved model is proposed. At the same time, the medical information system applying the improved model is designed according to the complex actual needs. The purpose of this paper is to correctly understand the positive role of medical sports big data (BD) research in the medical field and standardize the behavior of medical staff. On the one hand, it can improve the safety awareness of patients and enhance the standardization of medical treatment environment. This paper will analyze the meaning and research status of medical data from the perspective of legal risk control, focus on the status quo and existing problems of medical sports data privacy protection, and put forward positive countermeasures and some practical solutions. The results show that the medical sports information data has certain regularity and particularity, ease to spread, and mining. Hospitals and medical staff should make the areas and items restricted by law clear, standardize their own behaviors, constantly sum up experience, and actively improve and modify relevant measures.

## 1. Introduction

With the advent of the information age in the 20th century, the impact of information on the entire society has gradually increased to an absolutely important position [1, 2]. The speed of information dissemination and processing, the degree of application of information, and the amount of information are all rapidly increasing in a geometric progression. The medical information system stores a large amount of information about patients and hospitals. This information is huge and vital [3, 4].^l^ Once leaked, it may damage the reputation of the hospital and may even affect the normal operation of the hospital; for the patient, it may damage the patient's reputation and may even endanger the patient's life. Therefore, in the medical information system, it is particularly important to reduce the leakage of medical privacy information and protect the privacy information [5, 6].

The article "Medical Sports Data Privacy Protection Method Based on Legal Risk Control" was published in 2021. Journal: J Healthc Eng.

Nowadays, BD technology, like computer technology, is a new technological revolution and the best helper to promote economic development and industrial upgrading all over the world. BD technology has been deeply integrated into our lives from a single technology. In the new era, all kinds of data are open to the public, and the amount of data has increased dramatically. The introduction of Internet Plus is a combination of the Internet of Things, artificial intelligence, and the latest BD technology applications. Medical sports based on cloud computing and data storage have promoted the rapid development of medical sports [7]. At the same time, attention must be paid to further strengthen medical care and protect patient privacy. With the rapid establishment of the medical sports BD platform, the integration of BD technology and the medical sports field is getting closer and closer. In the promotion of medical technology, the application of BD is becoming more and more important. Therefore, the use of new technologies to develop our medical industry is a combination of not only time and tradition but also their common progress, mutual promotion, and complementarity.

The essence of BD is massive data, but it is not the only feature of BD. The BD technology of medical and sports industry is based on the traditional data accumulation and existing medical sports technology, combined with some new data analysis technology and high-speed communication technology [8, 9]. With BD and mobile Internet technology and the popularity of related medical and sports wearable devices, ordinary people can wear medical and sports equipment in daily life or collect a large number of physical signs and related user information through other near-field biological sign sensors. The network obtains real-time, continuous disease diagnosis or health services from the medical sports diagnosis platform or health service platform and truly realizes the continuous monitoring of health information by users anytime and anywhere. However, in the actual diagnosis process, the interactive data between the participating entities usually contain some sensitive information of the participating entities. At present, there are no specific and reasonable implementation methods for the protection of sensitive personal information of users or patients. How to correctly face the problems and explore the countermeasures is an urgent task for academic researchers. The research on privacy protection mainly focuses on two aspects: one is the privacy protection of training data used in the training process of classification model [10]; the second is the privacy protection of classification data and classification model parameters in the process of using classification model to treat classified data. Generally speaking, experts and scholars focus on the importance of medical and sports BD, most of which are concentrated in the analysis of overall advantages. There are few researches on specific implementation measures, especially the use of BD technology to distinguish between sharing results and leaking patients' privacy. Secondly, the development status of medical sports BD is analyzed. There are more researches in the field of medical and sports, and comprehensive research is conducted from the system and policy to the innovation and reform ability of enterprises [11, 12]. Foreign scholars should increase the research on medical sports BD problem solving, carry out more in-depth analysis of the problems, put forward feasible strategies, combined with the current economic development situation and the needs of patients, and explore a new path for the healthy development of medical and sports BD.

The article "Medical Sports Data Privacy Protection Method Based on Legal Risk Control" was published in 2021. Journal: J Healthc Eng.

This paper starts with the meaning and characteristics of BD, explores the development status of BD of medical sports, and elaborates the characteristics and types of medical sports BD and its application in medical sports and health field. It mainly analyzes the problems of the protection of personal privacy of medical sports BD, finds out the reasonable use method and the balanced basis point in line with the characteristics of BD, and organically analyzes the two aspects. This paper will classify and discuss the privacy protection challenges that may be faced in the application of medical sports BD privacy protection system and legal risk control theory under BD and make plans from objective and subjective aspects, respectively, and make objective outlook on the development direction. It hopes to provide theoretical basis for medical sports workers to meet problems, innovate management mode, and clear the direction of solution. The paper analyzes the current citation mode and studies foreign experience. Through comparative advantage analysis, it concludes the similarities and differences of domestic use of medical sports data development, learning advanced experience, proposing improved methods and paths, and combining with new development methods; finally, it puts forward a new model of BD development in medical sports field in China.

## 2. BD and Privacy Protection in Medical Sports Field

### 2.1. The Concept and Significance of BD

In terms of clinical medical diagnosis, due to the large individual differences between different patients, similar conditions may have very different causes. Doctors need to spend energy to communicate and check face-to-face with each patient before they can give a diagnosis. However, since the doctor may be affected by previous experience in the diagnosis or omission of the patient′s examination, various reasons may cause misdiagnosis, especially some intractable diseases. The use of big data analysis can solve this problem well. Through the classification and sorting of a large amount of clinical diagnosis case data, the diagnosis model is constructed to provide doctors with auxiliary diagnosis results and improve the efficiency and accuracy of diagnosis. Of course, there are pros and cons in everything. Quantification, wide dissemination, and publicity of data have brought about many negative impacts on human society. The operation, management, collection, and processing of big data will have a certain impact on the protection of national privacy. According to the principle of “Privacy First” in government information management, we need to look at big data technology dialectically and seek advantages and avoid disadvantages, so as to meet the development requirements of society.

The article "Medical Sports Data Privacy Protection Method Based on Legal Risk Control" was published in 2021. Journal: J Healthc Eng.

In this society, advanced science and technology, information circulation, and people's communication are becoming closer and more convenient, and BD is the product of this high-tech era. The future era is not the IT era but the DT era. DT is a data technology, which shows the importance of BD. Compare the data with a vibrant coal mine. Coal is divided into coking coal, anthracite coal, fatty coal, and lean coal according to its properties, but the drilling costs of open-pit mines and deep-mount mines are different. Similarly, BD is “convenient” rather than “large.” Value content and mining costs are more important than quantity. For many industries, how to use these large amounts of data is the key to winning the competition. The value of BD is reflected in the following aspects. Companies that provide products and services to a large number of consumers can use big data for accurate marketing. Long-tail companies that manufacture small American models can use big data for service conversion. Traditional companies that must change under the pressure of the Internet need to keep pace with the times; and make full use of the value of big data. However, the importance of “BD” in economic development does not mean that it can replace all rational thinking about social issues. A large amount of data cannot eliminate the logic of scientific development. The famous economist Ludwig von Mises has issued the following warning: “Today, many people are busy accumulating useless information and cannot understand its special economic importance by explaining and solving problems.”

The article "Medical Sports Data Privacy Protection Method Based on Legal Risk Control" was published in 2021. Journal: J Healthc Eng.

But big data technology brings about not only convenience to our lives but also the risk of privacy data leakage. In recent years, privacy leaks have occurred continuously, and, because of the high degree of privacy of medical data, the privacy protection issue in medical data processing is more important. Compared with other data information, once the user's medical data is leaked, it will cause serious and irreparable harm to the user and the society. Therefore, we need to be extra cautious when using big data to process medical data. Organizations can use relevant data and analysis to reduce costs, improve efficiency, develop new products, and make more informed business decisions. Combining big data with high-performance analytics, companies can analyze the root causes of failures, problems, and defects in a timely manner, save billions of dollars each year, and plan real-time traffic routes for thousands of high-speed vehicles. You can avoid congestion and analyze all SKUs and prices. Then clear the inventory to get the maximum profit. According to customers' buying habits, increase the priority of interest, quickly identify golden customers from a large number of customers, and use click stream analysis and data mining to avoid fraud.

### 2.2. The Meaning and Characteristics of Big Medical Sports Data

People have achieved unprecedented contact through the Internet of things, which is thousands of miles away. Besides, we can communicate with each other through the Internet. BD positioning analysis can help us better choose our own suitable direction and provide diversified personalized services to solve the problems around us. However, at the same time, it also leads to the risk of personal privacy leakage. Privacy issues are more important in the field of medical sports. Medical and sports institutions inevitably use the patient's medical record data in the process of scientific research and diagnosis.

Because the individual differences of different patients are very large, similar conditions may have very different causes. Doctors need to spend energy to communicate and check face-to-face with each patient before they can give a diagnosis. However, since the doctor may be affected by previous experience in the diagnosis or omission of the patient′s examination, various reasons may cause misdiagnosis, especially some intractable diseases. The use of big data analysis can solve this problem well. Through the classification and sorting of a large amount of clinical diagnosis case data, the diagnosis model is constructed to provide doctors with auxiliary diagnosis results and improve the efficiency and accuracy of diagnosis.

The article "Medical Sports Data Privacy Protection Method Based on Legal Risk Control" was published in 2021. Journal: J Healthc Eng.

Therefore, it is necessary to collect and release the medical sports data of some patients within a certain period of time. However, in this process, the patient's privacy information is easy to be leaked, which will not only play a side effect on the improvement of the patient's condition but also may cause indelible damage to the patient's psychology. At present, with the combination of medical sports and BD, high medical costs, and tense doctor-patient relationship, people are paying more and more attention to privacy protection in the fields of medicine and sports. Data privacy protection technology is especially important, because if you only rely on laws, regulations, and human norms, you cannot achieve effective constraints. BD technology has produced subtle influences and changes in the medical field. Due to the current state of the medical exercise data in the BD environment, the medical exercise BD is characterized by a large amount of medical data, the wide application of electronic medical records, and the expansion of the data collection range. First, there is a large amount of medical and sports data. BD is a huge amount of data. Living conditions in our country are constantly improving, and the average life expectancy is steadily increasing. The important reason is that the medical and sports health conditions are constantly improving, and the national medical and sports field has always been constantly innovating and improving the conditions. The collection of medical and sports data has a large amount and many kinds and involves a wide range. Further deepening will improve the medical service ability and work efficiency of the hospital.

### 2.3. Privacy Protection of Big Medical Sports Data

Medical diagnoses by, for example, hospitals are trusted by patients. When patients go to the hospital, they must provide the most detailed information for the doctor, which is conducive to the doctor's judgment of the condition and timely treatment in the future. When patients fill in medical records or basic information, the relationship between patients and doctors is the particularity of mutual trust. Patients elaborate on their physical condition and disease characteristics. Therefore, the patient's disease characteristics and personal characteristics will appear in the medical records, and this information contains the privacy information about the patient. This information is limited to attending physicians and related personnel in order to cure the disease. If the information related to medical records is unfortunately leaked, it will seriously violate the dignity and personality of patients. During the patient's visit to the hospital, the doctor chooses the appropriate treatment according to the patient's condition and personal characteristics. In this process, a lot of patient information is generated. For example, the patient's name, age, marital status, genetic history, and other information not only reflect the various examinations and physical conditions of each patient in hospital but also reflect the personal information and related life characteristics of the patient, for example, the patient's eating habits, whether the patient's organ system is different from the ordinary patients, and so on. A detailed medical record contains all kinds of information about the patient which can reflect the patient's current physical condition and living conditions and has the value that doctors and patients cannot ignore. But this value can only be fully highlighted on the basis of ensuring that medical information can be protected.

The article "Medical Sports Data Privacy Protection Method Based on Legal Risk Control" was published in 2021. Journal: J Healthc Eng.

At present, in the formal and legal medical diagnosis platform, some reasonable methods are used to protect patient privacy. In the treatment of patients, the distinctive and prominent signs such as name, age, and ID number represent personal privacy. Without affecting the accuracy of information, data security can be guaranteed by anonymous processing of this information. In practice, researchers and medical experts have also explored data identification deletion before the publication of the identification and then anonymous processing of the data. In this way, the accuracy of the diagnosis process can be guaranteed on the basis of privacy protection. In the specific implementation process, data problems can also be dealt with in a way of lossy links and generalizations to ensure the integrity of medical data. Among the numerous medical data, the importance and priority of information are different. If we adopt a high-intensity privacy protection measure for all medical data, we will not only fail to distinguish the importance of data but also increase the cost and waste resources. Therefore, some foreign hospitals and health treatment and rehabilitation platforms adopt the hierarchical protection system of medical data, not only for the core data but also for different levels of information data. Therefore, we should constantly improve the data privacy protection technology of medical information, so that the privacy of medical patients in China cannot be violated. In the information networking system in the medical field, the entry threshold is low, the number of participants is large, and the ways of data leakage are various. Therefore, access control technology is used to set different access rights for different staff members, which can also objectively promote the classification of medical data. At the same time, it can be classified in content to improve the efficiency of inquiry. However, in the current technical design, the specific process and means are complex and diverse. There are no unified design rules to standardize the unified access rules. In some cases, there are special information data that need to be processed separately, and the overall management and adjustment are not complete. Therefore, in the privacy protection of medical data, it is necessary to strengthen the research on rule setting and find and overcome technical difficulties.

The article "Medical Sports Data Privacy Protection Method Based on Legal Risk Control" was published in 2021. Journal: J Healthc Eng.

## 3. Privacy Protection of Medical Sports Data under Legal Risk Control

### 3.1. Ways of Data Privacy Leakage

With the development of information technology, privacy leakage is happening. With the development of information technology, data and information left over from the Internet are connected through computers and mobile terminals. Patient data is leaked through the Internet. Vulnerabilities include access environment and transmission network. Disclosure of the privacy of the hepatitis B virus bank will lead to discrimination in job hunting, and the potential illness of patients will be leaked out, resulting in mental stress and even depression. Many privacy leaks occur without the knowledge of the parties. Some companies deliberately collect personal privacy on the network or illegal intrusion into the database of some medical institutions to steal data, even if these leaked data are not directly used, causing losses to the parties, and even the records have been deleted. This situation should also belong to the problem of medical data security, which may have potential hazards and should be paid attention to. In addition to the above, there are many channels for medical data leakage. Some nonprofit personnel seek tampering with data orientation, fishing attacks, and other ways to obtain the collected data in the process of information acquisition and sell them through reselling and transferring. With the combination of BD and mobile Internet of Things, the network is frequently used and the security is greatly reduced. In the context of linking Wi-Fi, when the medical information collector uploads the collected data, the attacker can use deception to tamper with the address of the upload server, which leads to the direct transmission of medical information to the server designated by the attacker. Let the hospital take precautions. In the process of data storage after information collection, attackers decrypt and analyze the data by intercepting the encrypted information in the transmission process, retrospectively store the server address, and obtain attribute data. After obtaining a large amount of data, the AI analysis is carried out to compare the user's personal data, such as location information, browsing records, communication mode, and server data, and ultimately obtain privacy information. In the process of extracting personal information, after the attacker intercepts the information, the analysis and comparison of useful information such as height, inquiry record, and location service can result in the second leakage of user privacy data. Therefore, data privacy protection measures for medical information are prescribed to prevent leakage by limiting output, data, and access. The survey of privacy protection of patients is shown in Table 1.

The article "Medical Sports Data Privacy Protection Method Based on Legal Risk Control" was published in 2021. Journal: J Healthc Eng.

### 3.2. Privacy of Legal Risk Control

From the legal point of view, the patient's electronic medical record contains a lot of personal privacy information, which involves many aspects of the patient's life, including diagnosis results, real-time information in the treatment process and the patient's own health status, and genetic and other related privacy information. In recent years, patients at home and abroad are also very concerned about the privacy protection of personal medical data, so many countries have gradually established privacy protection laws. In 1974, the Privacy Act was established in the United States to protect the privacy of individual citizens. This law developed into the basis of privacy protection. In 1996, the U.S. Congress introduced HIPAA, which enacted detailed legal stripes and regulations for medical information, enabling patients privacy and detailed medical data to be fully protected, which is another progress in the privacy protection of large medical data. In the 21st century, HHS further developed the Privacy Standard of Personal Recognizable Health Information according to the specific content of HIPAA. So far, the United States has established a relatively perfect legal system to protect the privacy of patients' medical data; and its laws are operable. The BD of medical treatment under the protection of law is guaranteed. If there is abuse of privacy profit, it will be punished by law. Our country pays less attention to patient privacy protection, and there is no perfect system to protect it. Privacy protection laws for patients' medical information are rarely mentioned in Nurse Management Law, Licensed Physicians Law, and Regulations on AIDS Monitoring and Management. On August 30, 2017, the National Information Security Standardization Technical Committee issued the Guidelines for the Assessment of Information Technology Safety Data Exit Safety (Draft). It identified personal electronic medical records, health records, and other population information as important data. At present, our country's science and technology are not developed enough to effectively promote electronic medical records. Secondly, in the sharing and use of medical information, medical units and related units have not reached agreement, so it is impossible to formulate appropriate reasonable standards. At the same time, our national awareness of data privacy protection of medical information is not enough. When patients have privacy leaks and medical disputes, they cannot effectively protect their rights and interests. Therefore, we should speed up the construction of legal system, so that medical platforms can make use of the rights granted by law to avoid or reduce the adverse consequences of legal risks.

The article "Medical Sports Data Privacy Protection Method Based on Legal Risk Control" was published in 2021. Journal: J Healthc Eng.

## 4. Problems and Protection Methods of Medical Sports Data Privacy

### 4.1. Problems in Privacy of Medical Sports Data

1. The particularity of medical sports data. Medical sports BD is different from other business data because of its strong privacy and contains more personal information of patients, so it derives special sensitivity and importance. So many people do not realize the particularity of medical sports data. The reasons for medical data privacy leakage are shown in Figure 1.
2. The ownership of medical sports data is unknown. In some regions, the unclear ownership of personal information privacy is the cause of disputes. Some patients believe that medical sports data reflect the health status of patients and other personal information should belong to patients. The boundary of the right to use and keep the patient's medical record is vague. As shown in Figure 2, almost every kind of information belongs to both sides of the same argument.
3. Privacy protection technology is not good. In today's highly developed network, network technology security is very important. Due to poor awareness of prevention, low protection technology, hackers' attack, and access to medical sports data and patient's personal information, some medical sports diagnosis platform database even has no basic firewall settings.

### 4.2. Privacy Protection Method of Medical Sports Data

According to the data analysis of the experiment, the importance ratio of the medical and sports data privacy protection method can be obtained as shown in Figure 3.

1. The premise is to respect the privacy of others. From a moral point of view, respect for the privacy of others is a criterion that everyone should abide by, especially in the privacy protection of medical and sports data in the environment involving BD. The use of BD and the Internet of things has changed the relationship between medical research and practice and has also created new security challenges in terms of privacy protection. Patients' privacy information is easier to collect and disseminate, so it is essential to respect others' privacy while applying BD. In some disease analysis, according to patient privacy and pathological data, through BD matching and analysis, it is very easy to infer the living habits and occupational characteristics. Therefore, as a medical worker, we should not disclose the patient's privacy and disease situation to the outside world. We should respect and protect the privacy of the patient, and we should not make use of this information for profit.
2. Establish and improve relevant laws and regulations. In terms of system and policy, establishing and perfecting relevant laws and regulations are the key link of medical data privacy protection. The protection of medical sports privacy has become a key factor in the doctor-patient relationship. The right of privacy of patients is given to patients by law when they receive medical and sports services. If they are illegally disclosed for profit, they will be severely punished in accordance with the law. The privacy protection of medical and sports data should focus on BD legislation to ensure the security of personal information and make the use of BD more standardized. At the legislative level, to block the black hole of data privacy, we should strengthen the comprehensiveness, systematicness, and specialization of laws and regulations and crack down on the behavior of lending, leasing, and reselling personal privacy. It is also necessary to establish a targeted personal information protection law to promote the reasonable flow of health, medical, and sports data according to law.
3. Improve information privacy protection technology. Improving information privacy protection technology is the technical supplement of medical and sports BD technology. As a necessary condition of privacy protection, technology can avoid the leakage of medical and sports data to a certain extent. In the stage of data collection, if anonymization is adopted, it can be very effective in various methods of restricting data, and its application is also more extensive. As shown in Figure 4, online hierarchical medical sports diagnosis system can effectively provide protection mechanism. At the same time, strengthening and improving the identifier processing technology can effectively avoid data leakage and protect sensitive information in the data.

The article "Medical Sports Data Privacy Protection Method Based on Legal Risk Control" was published in 2021. Journal: J Healthc Eng.

## 5. Conclusion

This paper briefly analyzes the problems and countermeasures of medical and sports data privacy protection under the background of BD and legal risk control. In the environment of rapid development of modern economy, the new opportunities and problems of medical sports BD, personal privacy, and medical and sports achievements were expounded. The application of medical sports BD is a new trend in the field of medical sports. This paper points out that, under the opportunity of Internet BD blowout development, changing the traditional treatment sports mode, grasping the law, exploring the new role of Internet application, and correctly understanding and solving the problems of medical sports BD mode are the key breakthrough to promote the development of medical sports field in the new era.

This paper introduces the current situation of medical and sports data utilization in China and the ways and classification of privacy protection, combines the cost of legal risk control, and analyzes the status mode of traditional medical sports governance. Combined with the characteristics and essential characteristics of BD and the experience and lessons at home and abroad, this paper puts forward a new way out and development power to explore the legal role of market supervision and promote the growth of medical and sports industry.

Big data not only brings about convenience to people′s life but also brings about the risk of privacy information leakage. Medical information system is a more complex system, which has certain dynamics and flexibility. This method can greatly improve the construction speed of the system database. It can not only solve the problem of privacy leakage in the medical environment but also improve the existing medical environment.

## Figures and Tables

**Figure 1:** Reasons for medical data privacy leakage.

**Figure 2:** Proportion of sponsor′s opinion on medical data.

**Figure 3:** Proportion of importance of medical sports data privacy protection methods.

**Figure 4:** Model diagram of online graded medical diagnosis system.

**Table 1:** Survey of privacy protection of patients.

Type	Number
Number of inpatients	6232
Level 1 privacy leakage	4215
Level 2 privacy leakage	1268
Registered electronic medical record	5998
Valuable medical record data	2055

## Data Availability

No data were used to support this study.

## References

[1] Kumar A. (2019). Design of secure image fusion technique using cloud for privacy-preserving and copyright protection. *International Journal of Cloud Applications and Computing*.

[2] Kai F., Wei J., Hui L., Yang Y. (2018). Lightweight rfid protocol for medical privacy protection in iot. *IEEE Transactions on Industrial Informatics*.

The article "Medical Sports Data Privacy Protection Method Based on Legal Risk Control" was published in 2021. Journal: J Healthc Eng.

[3] Chen F., Luo Y., Ji Z., Zhu J., Zhang Z., Zhao C. (2017). An infrastructure framework for privacy protection of community medical Internet of things. *World Wide Web-Internet & Web Information Systems*.

[4] Takaiigarashi T., Kinoshita K., Nagasaki M., Ogishima S., Nakamura N., Nagase S. (2017). Security controls in an integrated biobank to protect privacy in data sharing: rationale and study design. *Bmc Medical Informatics & Decision Making*.

[5] Sarabdeen J., Moonesar I. A. (2018). Privacy protection laws and public perception of data privacy. *Benchmarking: An International Journal*.

[6] Sher M.-L., Talley P. C., Cheng T.-J., Kuo K.-M. (2017). How can hospitals better protect the privacy of electronic medical records? Perspectives from staff members of health information management departments. *Health Information Management Journal*.

[7] Parvees M. Y. M., Samath J. A., Raj I. K., Nirmal R. M. (2017). Chaos-based steganocryptic approach to protect medical images with text data of patients. *Journal of Medical Imaging and Health Informatics*.

[8] Yamada H., Inoue Y., Shimokawa Y., Sakata K. (2017). Skin stiffness determined from occlusion of a horizontally running microvessel in response to skin surface pressure: a finite element study of sacral pressure ulcers. *Medical & Biological Engineering & Computing*.

[9] Liyanage H., Liaw S.-T., Konstantara E. (2018). Benefit-risk of patients′ online access to their medical records: consensus exercise of an international expert group. *Yearbook of Medical Informatics*.

[10] Reichel J. (2017). Oversight of EU medical data transfers - an administrative law perspective on cross-border biomedical research administration. *Health and Technology*.

[11] Wamba S. F., Gunasekaran A., Papadopoulos T., Ngai E. (2018). Big data analytics in LoGistics and supply chain management. *International Journal of Logistics Management*.

[12] Napoli C., Pappalardo G., Tramontana E., Zappalà G. (2018). A cloud-distributed gpu architecture for pattern identification in segmented detectors big-data surveys. *Computer Journal*.

